# New Claims for Wild Carrot (*Daucus carota* subsp.* carota*) Essential Oil

**DOI:** 10.1155/2016/9045196

**Published:** 2016-02-14

**Authors:** Jorge M. Alves-Silva, Mónica Zuzarte, Maria José Gonçalves, Carlos Cavaleiro, Maria Teresa Cruz, Susana M. Cardoso, Lígia Salgueiro

**Affiliations:** ^1^Faculty of Pharmacy, University of Coimbra, Azinhaga de S. Comba, 3000-354 Coimbra, Portugal; ^2^Center for Neuroscience and Cell Biology, University of Coimbra, 3004-517 Coimbra, Portugal; ^3^Faculty of Medicine, University of Coimbra, Azinhaga de S. Comba, 3000-548 Coimbra, Portugal; ^4^Department of Chemistry & QOPNA, University of Aveiro, 3810-193 Aveiro, Portugal

## Abstract

The essential oil of* Daucus carota* subsp.* carota* from Portugal, with high amounts of geranyl acetate (29.0%), *α*-pinene (27.2%), and 11*α*H-himachal-4-en-1*β*-ol (9.2%), was assessed for its biological potential. The antimicrobial activity was evaluated against several Gram-positive and Gram-negative bacteria, yeasts, dermatophytes, and* Aspergillus* strains. The minimal inhibitory concentration (MIC) and minimal lethal concentration (MLC) were evaluated showing a significant activity towards Gram-positive bacteria (MIC = 0.32–0.64 *μ*L/mL),* Cryptococcus neoformans* (0.16 *μ*L/mL), and dermatophytes (0.32–0.64 *μ*L/mL). The inhibition of the germ tube formation and the effect of the oil on* Candida albicans* biofilms were also unveiled. The oil inhibited more than 50% of filamentation at concentrations as low as 0.04 *μ*L/mL (MIC/128) and decreased both biofilm mass and cell viability. The antioxidant capacity of the oil, as assessed by two* in chemico* methods, was not relevant. Still, it seems to exhibit some anti-inflammatory potential by decreasing nitric oxide production around 20% in LPS-stimulated macrophages, without decreasing macrophages viability. Moreover, the oils safety profile was assessed on keratinocytes, alveolar epithelial cells, macrophages, and hepatocytes. Overall, the oil demonstrated a safety profile at concentrations below 0.64 *μ*L/mL. The present work highlights the bioactive potential of* D. carota* subsp.* carota* suggesting its industrial exploitation.

## 1. Introduction

Aromatic and medicinal plants, such as those found in Lamiaceae and Apiaceae families, have been widely used in folk medicine to treat several ailments. Their effects are particularly associated with the essential oils, which are widely described as having several bioactive properties such as antioxidant, anti-inflammatory, antifungal, and antibacterial ones [1–3].

Plants of the genus* Daucus* L. (Apiaceae) grow mostly in temperate regions of Europe, West Asia, and Africa. Nevertheless, some species have been found to grow in North America and Australia [4, 5]. The species* Daucus carota* L., commonly known as carrot, is recognized worldwide due to its roots widely used for both food and medicinal purposes [6]. In addition, the seed essential oil has also been described as antihelmintic, antimicrobial, hypotensive, and diuretic, amongst other biological properties [4].

This taxon includes eleven highly polymorphic, interrelated, and interhybridized taxa [7–9], among which some have been widely studied with regard to their bioactive properties. Nevertheless, only a few studies identify the subspecies used, a very important aspect to consider bearing in mind the high variability mentioned. For example,* D. carota* subsp.* halophilus* essential oil has been reported for its antifungal properties against several human pathogenic fungi [7]. In turn, besides the antifungal activities,* D. carota* subsp.* gummifer* essential oil has also been described as an anti-inflammatory agent [10] while that of* D. carota* subsp.* maritimus* has been pointed out as exhibiting a potential antibacterial effect [11].

Regarding the subspecies* D. carota* subsp.* carota*, the antifungal effects of its essential oil were previously reported [12] and although a significant antifungal effect was claimed, the mechanism of action underlying such effects was not assessed. Therefore, in the present study, besides the antifungal effect of the oil against several yeasts (*Candida* strains,* Cryptococcus neoformans*), dermatophytes (*Trichophyton* spp.,* Epidermophyton*, and* Microsporum* spp.), and* Aspergillus* strains, we also aim to elucidate a possible mode of action particularly on* Candida albicans*. For that, the effect of the oil on the inhibition of the germ tube formation, an important virulence factor, as well as the effect of the oil on preformed biofilms, was considered. Additionally, other biological properties of the essential oil were also evaluated, namely, the antibacterial, antioxidant, and anti-inflammatory properties, in order to identify a broader bioactive potential of the oil for its industrial exploitation. Moreover, considering the lack of cytotoxic studies on the essential oil of this subspecies and the putative interest to develop a plant-based product to be used on humans and/or animals, the safety profile of the essential oil against macrophages (Raw 264.7), keratinocytes (HaCaT), epithelial alveolar cells (A549), and hepatocytes (HepG2) was also evaluated.

## 2. Material and Methods

### 2.1. Essential Oil Isolation and Analysis

Ripe umbels with seeds of* D. carota* subsp.* carota* were collected at Serra da Lousã, Coimbra (Portugal), on the 1st of July 2013. A voucher specimen (Ligia Salgueiro 78) was deposited at the Herbarium of the Faculty of Pharmacy of the University of Coimbra. The essential oil was obtained by hydrodistillation from air dried umbels in a* Clevenger*-type apparatus according to the European Pharmacopoeia [13]. Oil analyses were carried out by gas chromatography (GC) and gas chromatography/mass spectrometry (GC/MS). GC was carried out on a Hewlett Packard 6890 gas chromatograph (Agilent Technologies, Palo Alto, California, USA) with HP GC ChemStation Rev. A.05.04 data handling system, equipped with a single injector and two flame ionization detectors (FID). A Graphpak divider (Agilent Technologies, part number 5021-7148) was used for simultaneous sampling in two Supelco (Supelco Inc., Bellefonte, PA, USA) fused silica capillary columns with different stationary phases: SPB-1 (polydimethylsiloxane; 30 m × 0.20 mm i.d., film thickness 0.20 *μ*m) and SupelcoWax-10 (polyethylene glycol; 30 m × 0.20 mm i.d., film thickness 0.20 *μ*m). Conditions were as follows: oven temperature program: 70–220°C (3°C/min), 220°C (15 min); injector temperature: 250°C; carrier gas: helium, adjusted to a linear velocity of 30 cm/s; splitting ratio 1 : 40; detectors temperature: 250°C. GC/MS analyses were performed on a Hewlett Packard 6890 gas chromatograph fitted with HP1 fused silica column (polydimethylsiloxane; 30 m × 0.25 mm i.d., film thickness 0.25 *μ*m), interfaced with Hewlett Packard Mass Selective Detector 5973 (Agilent Technologies, Palo Alto, CA, USA) operated by HP Enhanced ChemStation software, version A.03.00. GC parameters were as above; interface temperature was 250°C; MS source temperature was 230°C; MS quadrupole temperature was 150°C; ionization energy was 70 eV; ionization current was 60 *μ*A; scan range was 35–350 *μ*, with 4.51 scans/s [14]. The volatile compounds were identified by both their retention indices and mass spectra. Retention indices, calculated by linear interpolation relative to retention times of a series of* n*-alkanes, were compared with those of authenticated samples from the database of the Laboratory of Pharmacognosy of the Faculty of Pharmacy of the University of Coimbra. Mass spectra were compared with reference spectra from a home-made library or from literature data [15, 16]. Relative amounts of individual components were calculated based on GC peak areas without FID response factor correction.

### 2.2. Antibacterial Assays

The antibacterial activity of the oil was evaluated against Gram-positive strains (*Bacillus subtilis* ATCC 6633,* Listeria monocytogenes* CBISA 3183, and* Staphylococcus aureus* ATCC 6538) and Gram-negative ones (*Escherichia coli* ATCC 25922 and* Salmonella typhimurium* ATCC 14028). The minimal inhibitory concentrations (MICs) and the minimum lethal concentrations (MLCs) were assessed according to the Clinical and Laboratory Standards Institute (CLSI) reference protocol M07-A9 [17]. Briefly, serial doubling dilutions of the oil were prepared in dimethyl sulfoxide (DMSO, Sigma Life Science, Sigma-Aldrich, MO, USA) with concentrations ranging from 0.08 to 20 *μ*L/mL. Recent cultures of each strain were used to prepare the cell suspensions (1-2 × 10^5^ CFU/mL) and cell concentration was confirmed by viable count on Mueller Hinton Agar (Oxoid, Hampshire, England). All tests were performed using Mueller Hinton Broth medium and the test tubes were incubated aerobically at 37°C for 24 h and then MICs were registered. To evaluate MLCs, 20 *μ*L of broth was taken from each negative tube after MIC reading, cultured in Mueller Hinton Agar plates, and incubated as mentioned above. The sensitivity of tested strains was controlled by the use of a reference compound, ampicillin (Fluka BioChemika, Buchs, Switzerland). All tests were performed in duplicate. The MIC and MLC values were considered when three independent assays had the same value.

### 2.3. Antifungal Activity and Mechanism of Action Assays

The antifungal properties of the essential oil were tested against three* Candida* reference strains (*C. albicans* ATCC 10231,* C. tropicalis* ATCC 13803, and* C. parapsilosis* ATCC 90018) and two clinical strains (*C. krusei* H9 and* C. guilliermondii* MAT23); one* Cryptococcus neoformans* reference strain (*C. neoformans* CECT 1078); four dermatophyte strains (*Trichophyton rubrum* CECT 2794,* T. mentagrophytes* var.* interdigitale* CECT 2958,* T. verrucosum* CECT 2992, and* Microsporum gypseum* CECT 2908); the remaining dermatophytes were clinically isolated (*T. mentagrophytes* FF7,* M. canis* FF1, and* Epidermophyton floccosum* FF9); two reference* Aspergillus* strains (*A. niger* ATCC 16404 and* A. fumigatus* ATCC 46645); and one* Aspergillus* strain was from a clinical origin (*A. flavus* F44). The MICs and MLCs were assessed according to the CLSI reference protocols M27-A3 [18] and M38-A2 [19] for yeasts and filamentous fungi, respectively, as previously described by Zuzarte et al. [20].

To elucidate a possible mechanism of action underlying the antifungal effects, two assays were considered: the inhibition of* C. albicans* germ tube formation and the disruption of its preformed biofilms, in the presence of the essential oil. The first assay was tested as previously reported by Pinto et al. [21]. The percentage of germ tubes was determined as the number of cells showing hyphae at least as long as the diameter of the blastospore. Cells showing a constriction at the point of connection of the hyphae to the mother cell, typical for pseudohyphae, were excluded. Results are shown as mean ± standard deviation of three independent determinations. The effect of the essential oil on preformed* C. albicans* biofilm was evaluated using the method described by Taweechaisupapong et al. [22] with some modifications. Briefly, a loop of SDA culture of* C. albicans* grown for 24 h at 37°C was suspended in Yeast Peptone Dextrose (YPD) broth (1% yeast extract, 2% peptone, and 2% dextrose) and incubated for 24 h at 37°C. Then, cells were thoroughly washed twice with sterile PBS (pH 7.4) (0.8% NaCl, 0.02% KH_2_PO_4_, 0.31% Na_2_HPO_4_·12H_2_O, and 0.02% KCl). Between each washing step, the suspension was submitted to 10 min centrifugation at 3000 g. Cell density was adjusted to approximately 1 × 10^6^ CFU/mL, using a haemocytometer, and then 100 *μ*L of the final suspension was added to 96-well microtiter plates and incubated for 24 h at 37°C, to form the biofilms. Following three washing steps with PBS, the essential oils (1.25–10 *μ*L/mL, prepared in RPMI) were added and incubated for 24 h, at 37°C. Both negative and positive controls were considered using sterile RPMI broth and inoculated RPMI broth, respectively. Biofilm mass was quantified using crystal violet according to Raut et al. [23]. Biofilm viability was evaluated using the XTT assay, as described by Saharkhiz et al. [24] with some modifications. Briefly, after biofilm formation and treatment with essential oils, the medium was removed and biofilms were thoroughly washed with PBS. To a solution of XTT (1 mg/mL), menadione (10 mM in acetone) was added to a final concentration of 4 *μ*M. 100 *μ*L of this solution was added following incubation for 2 h at 37°C in the dark. The absorbance was observed at 490 nm and biofilm viability was determined by comparing the absorbance of treated samples with those of untreated ones. Results are shown as mean ± standard deviation of three independent determinations performed in duplicate.

### 2.4. Antioxidant Assays

The antioxidant properties of the essential oil were determined using two different antioxidant assays, namely, the 2,2′-azino-bis(3-ethylbenzothiazoline-6-sulfonic acid) (ABTS^•+^) scavenging and oxygen radical absorbance capacity (ORAC) assays. The ABTS^•+^ scavenging assay was performed according to the procedure described by Re et al. [25], with some modifications. Briefly, the ABTS^•+^ stock solution was prepared by the reaction of ABTS-NH_4_ aqueous solution (7 mM) with 2.45 mM dipotassium persulfate in the dark at room temperature for 12–16 h. This solution was then diluted until absorbance of 0.700 ± 0.03 at 734 nm. To determine the scavenging activity, 1 mL of ABTS^•+^ was added to 100 *μ*L of 0.64–20 mg/mL essential oil solution made in DMSO. After 20 min, the absorbance was read at 734 nm in a spectrophotometer against a blank (absolute ethanol). The antioxidant power of the samples was expressed as IC_50_ (*μ*g/mL) and compared to that of the standard compound, Trolox (0.75–12 *μ*g/mL). Data are shown as mean values ± standard deviation of three independent assays.

The ORAC assay was carried out using the method described by Garrett et al. [26] slightly modified. Briefly, 150 *μ*L of fluorescein (10 nM) was pipetted to a 96-well plate and 25 *μ*L of Trolox (25–200 *μ*M) or sample (0.32–10 mg/mL in phosphate buffer) was added. This mixture was incubated at 37°C for 10 min. After that, 25 *μ*L of 2,2′-azobis(2-amidino-propane) dihydrochloride (153 mM) was added to each well except that of negative control that contained 25 *μ*L of phosphate buffer. The fluorescence was immediately read on a plate reader every 1 min, in a total of 60 min. The emission wavelength was set at 530/20 nm and excitation wavelength at 485/20 nm. The area under the curve (AUC) was determined as described elsewhere [27]. The results, expressed as Trolox Equivalent (TE)/mg oil, are shown as mean ± standard deviation of at least three independent determinations.

### 2.5. Anti-Inflammatory Assay

The anti-inflammatory effect of the essential oil was determined through* in chemico* and* in vitro* assays using S-nitroso-N-acetyl-D,L-penicillamine (SNAP) as nitric oxide (NO) donor and through evaluation of NO release from lipopolysaccharide- (LPS-) stimulated macrophages, respectively.

For the* in chemico* assay, several concentrations of the oil (0.08–1.25 *μ*L/mL) were incubated with 0.9 *μ*L of the SNAP solution (100 mM) in endotoxin-free Dulbecco's Modified Eagle Medium (DMEM), in a final volume of 300 *μ*L, for 3 h. The NO scavenging activity was evaluated by quantifying nitrite levels in the medium using the Griess reaction, as previously mentioned [10]. For the* in vitro* assay, Raw 264.7, a mouse leukaemic macrophage cell line ATCC (TIB-71), was cultured in DMEM supplemented with 10% (v/v) non-inactivated foetal bovine serum, 3.02 g/L sodium bicarbonate, 100 *μ*g/mL streptomycin, and 100 U/mL penicillin at 37°C, in a humidified atmosphere of 95% air and 5% CO_2_. To evaluate the anti-inflammatory potential of the oil, macrophages (0.3 × 10^6^ cells/well) were cultured in 48-well microplates and allowed to stabilize for 12 h. Following this period, cells were either maintained in culture medium (control) or preincubated with different concentrations of the essential oil for 1 h and later activated with LPS (1 *μ*g/mL) for 24 h. Nitric oxide was quantified by measuring the accumulation of nitrites using the colorimetric Griess assay [28].

Simultaneously, cell viability was also determined using the resazurin method described by Riss et al. [29]. Metabolic active cells reduce resazurin (blue) into resorufin (pink) and therefore the magnitude of dye reduction is correlated with the number of viable cells. After the treatment described above for macrophages, resazurin solution (0.125 mg/mL) was added (1 : 10) and cells were further incubated at 37°C for 30 min in a humidified atmosphere of 95% air and 5% CO_2_. Quantification was performed using an ELISA microplate reader (SLT, Austria) at 570 nm, with a reference wavelength of 620 nm. A cell-free control was performed in order to exclude nonspecific effects of the oils on resazurin (data not shown).

### 2.6. Toxicological Profile

Cytotoxicity was evaluated in several mammalian cell lines, namely, human hepatocellular carcinoma cell line HepG2, ATCC number 77400; human keratinocyte cell line HaCaT, obtained from DKFZ (Heidelberg); human alveolar epithelial cell line A549, ATCC number CCL-185; and the mouse leukaemic monocyte macrophage cell line, previously mentioned.

Briefly, Raw 264.7 (0.6 × 10^6^ cells/mL), HepG2 (0.5 × 10^6^ cells/mL), HaCaT (0.2 × 10^6^ cells/mL), and A549 (0.2 × 10^6^ cells/mL) cell suspensions were prepared. Then, cells were cultured in 48-well microplates in a final volume of 600 *μ*L for 12 h and were further cultured with different concentrations (0.08 to 1.25 *μ*L/mL) of the essential oil, for 24 h. At the end, 60 *μ*L of resazurin (0.125 mg/mL) was added and the plates were then incubated for 30 min (Raw 264.7), 60 min (HepG2 and A549), and 120 min (HaCaT) at 37°C, in a humidified atmosphere of 95% air and 5% CO_2_. Cell viability was determined by reading the absorbance at 570 nm with a reference filter at 620 nm against a negative control (cells cultured in the absence of the oil) in an ELISA microplate reader (SLT, Austria). A cell-free control was performed in order to exclude unspecific effects of the oil on resazurin (data not shown).

### 2.7. Statistical Analysis

Data are expressed as mean ± standard error of the mean (SEM). Statistical significance was determined using one-way analysis of variance (ANOVA), followed by Dunnett's* post hoc* test. The statistical analysis was performed using Prism 5.0 Software (GraphPad Software). Differences were considered significant for *p* < 0.05.

## 3. Results and Discussion

### 3.1. Chemical Composition

The essential oil of* D. carota* subsp.* carota* was obtained from the umbels with a yield of 0.9% (v/w). Constituents of the oil are listed in Table 1, according to their elution order on a polydimethylsiloxane column. The oil is predominantly composed of hydrocarbon monoterpenes (46.6%) and oxygenated monoterpenes (29.5%), with geranyl acetate (29.0%) and *α*-pinene (27.2%) being the main components. Notably, these compounds were also identified as the main constituents of the essential oils obtained from flowering umbels of the same species grown in another region of Portugal (Cantanhede) [12], despite quantitative differences (37.9% for *α*-pinene and 15.0% for geranyl acetate). In turn, in opposition to that study, the* D. carota* subsp.* carota* oil herein obtained had a significant amount of oxygen containing sesquiterpenes (15.6%* versus* 2.5–3.1%), with 11*α*H-himachal-4-en-1*β*-ol being the main compound. This constituent was also identified as one of the main compounds in* D. carota* subsp.* carota* oil from plants of Italian origin [12].

### 3.2. Antibacterial Activity

The antibacterial potential of the oil against both Gram-positive strains (*Bacillus subtilis*,* Listeria monocytogenes*, and* Staphylococcus aureus*) and Gram-negative ones (*Escherichia coli* and* Salmonella typhimurium*) is summarized in Table 2. The results show that the oil was significantly more effective against Gram-positive bacteria, with MIC values in the range of 0.32–0.64 *μ*L/mL. Differences observed between Gram-positive and Gram-negative bacteria are mainly due to their distinct cell wall structure, as the cell wall of Gram-negative bacteria is much more complex comprising an outer membrane composed of hydrophilic polysaccharides chains that act as a barrier for hydrophobic essential oils [30].

Previously, the antibacterial activity of essential oils from the herb, flowering, and mature umbels of wild carrot growing in Poland was also tested [9]. Although direct comparisons between that study and the present one cannot be considered since a different antibacterial test was used (agar dilution method* versus* macrodilution broth method), the oils obtained in the previous work were much less effective against Gram-positive bacteria (MIC = 3–5 *μ*L/mL). These differences might be explained by distinct chemical compositions (*α*-pinene and sabinene* versus α*-pinene and geranyl acetate), as it is known that sabinene is devoid of antibacterial activity [31]. Instead, the essential oil herein used was primarily rich in geranyl acetate and *α*-pinene. These compounds have been tested for their antibacterial potential and several studies have pointed out the high antibacterial activity of *α*-pinene [32, 33] and weak activity of geranyl acetate [30], which may justify the activity of the oil. Nevertheless, minor compounds may also interfere with the antibacterial activity, and their potential effect should not be discarded.

### 3.3. Antifungal Activity and Mechanisms of Action

The antifungal activity of the essential oil against human and animal pathogens is presented in Table 3. In general, the oil was more effective against* Cryptococcus neoformans* (MIC = 0.16 *μ*L/mL) and dermatophyte strains, with MICs ranging from 0.32 to 0.64 *μ*L/mL. Regardless of the oil being much less effective against* Candida* spp. and* Aspergillus *spp., it showed a very low MIC for* C. guilliermondii*, similar to that found for dermatophytes (0.32 *μ*L/mL), thus suggesting some specificity of the oil for this strain. Overall, the oil showed both fungistatic and fungicidal effects against most of the strains tested since the MIC values were similar to MLC ones. Of note is the fact that the main isolated compounds identified in the oil herein studied, namely, geranyl acetate, *α*-pinene, and limonene, have also been previously assessed for their antifungal potential. Geranyl acetate demonstrated good antifungal effects against dermatophytes and* Cryptococcus neoformans*; however, it had a weak performance in inhibiting the growth of* Candida *strains and* Aspergillus *spp. [2, 21]. Similarly, *α*-pinene showed inhibitory effects against* C. albicans* and* Cryptococcus neoformans* [34, 35] as well as a potent effect against dermatophyte strains [36]. Moreover, Pinto et al. [21] also demonstrated that this compound exhibits a strong fungistatic and fungicidal activity, with this effect being preeminent for* Candida* and* Aspergillus* spp. Several authors have also described the antifungal activity of limonene against several fungi strains [36–39]. Therefore, the activity of these major compounds of* D. carota* subsp.* carota* essential oil may be responsible for the higher antifungal effects of this oil.

Although studies on the antifungal activity of* D. carota* subsp.* carota* oil were previously carried out, the mechanism of action underlying this effect remains unknown. Therefore, in the present study, we attempt to elucidate possible modes of action on* C. albicans*. For that, two assays were selected, namely, the inhibition of germ tube formation and the disruption of preformed biofilms.

The effects of subinhibitory concentrations of the essential oil on the inhibition of* C. albicans* germ tube formation are presented in Table 4. The oil was able to achieve more than 50% of filamentation inhibition at concentrations as low as 0.04 *μ*L/mL (MIC/128). This is quite interesting, since filamentation (dimorphic transition from yeast to filamentous form) in* C. albicans* is essential for virulence [40] and it seems that filamentation inhibition* per se* is sufficient to treat disseminated candidosis [41]. The striking difference between MICs and filamentation-inhibiting concentrations seems to suggest that different mechanisms of action may be responsible for these two biological effects. Geranyl acetate, the major compound of* D. carota *subsp.* carota* oil, may be responsible for this activity as assessed by Zore et al. [42]. This compound was highly effective against serum-induced morphogenesis (yeast to hyphal form transition in* C. albicans* ATCC 10231) with only 73 *μ*g/mL causing 63% inhibition of germ tube induction [42].

Figures 1 and 2 represent the effect of the essential oil on preformed* C. albicans* biofilms. The crystal violet method quantifies the biomass of the biofilm by staining it with the dye whereas the XTT assay evaluates cell viability by analysing the formation of a water soluble crystal formed after mitochondrial metabolization. Results show that the oil promoted a decrease of the biofilm biomass even for the lowest concentrations tested (Figure 1). Therefore, the results showed that the oil was able to interfere with preformed biofilms by reducing the amount of the attached biomass. Regarding biofilm cells viability, concentrations higher than 1.25 *μ*L/mL also reduced cell viability (Figure 2), compromising biofilm development. Note that the biofilm formation is a survival mechanism, contributing to microbial virulence and persistence [43, 44] since biofilms are very difficult to eliminate due to their high antifungal resistance in comparison to free-living cells. These results highlight the promising antibiofilm activity paving the way for future translational research on the treatment of disseminative candidiasis.

### 3.4. Antioxidant Analysis

The antioxidant analysis of the essential oil was carried out using the ABTS^•+^ scavenging and ORAC assays.  Table 5 summarizes the results obtained. It was seen that the essential oil is neither a good scavenger of ABTS^•+^ (IC_50_ = 1924.25 *μ*g/mL) nor a good peroxyl-induced oxidation inhibitor (ORAC values of 7.13 *μ*mol/TE/mg oil). Comparison of the present results with others for the same plant species is not possible due to the absence of the latter.

### 3.5. Anti-Inflammatory Activity

Chemical NO scavenging is a method possessing two valences; that is, it allows to evaluate the antioxidant potential of the essential oil by testing its ability to arrest this radical but also allows preliminary screening of the anti-inflammatory potential, since NO is a crucial mediator in inflammation.  Figure 3 summarizes the NO scavenging activity of the essential oil. The results showed that the essential oil had no scavenging activity towards NO for all the tested concentrations (0.08–1.25 *μ*L/mL). In order to deeply explore whether the essential oil modulates NO production, we also used an* in vitro* model of inflammation consisting of macrophages stimulated with* Toll-like* receptor 4 agonist LPS. Figures 4(a) and 4(b) summarize the NO release and the cell viability of LPS-stimulated macrophages treated with different concentrations of the essential oil, respectively. As far as we know, this is the first report on the anti-inflammatory activity of* D. carota* subsp.* carota*. As shown in Figure 4(a), incubation of macrophages with LPS, for 24 h, resulted in a significant increase in nitrite production. Taking into account the toxicity of the oil presented in Figure 4(b), inhibition of NO production was only considered for nontoxic concentrations of the oil. Indeed, NO production decreased by 19.04%, relatively to LPS (*p* < 0.05), without affecting cell viability in the presence of 0.64 *μ*L/mL of the oil. These results suggest a potential anti-inflammatory effect of the oil. Nevertheless, further experiments on different proinflammatory mediators and signal transduction pathways should be considered to confirm this activity.

The essential oil's major compounds, namely, geranyl acetate and *α*-pinene, may account for most of the oil's anti-inflammatory potential since previous studies have pointed out their anti-inflammatory potential (e.g., [45–47]).

### 3.6. Toxicological Profile

The cytotoxicity of the essential oil was screened in several mammalian cells lines in order to evaluate a potential pharmacological application of* D. carota* subsp.* carota* essential oil and the gathered results are summarized in Table 6. It can be inferred that the concentration of 0.64 *μ*L/mL induces different cell viability results among all the cell lines studied, with macrophages being the most resilient (92.83% ± 1.04 cell viability) and hepatocytes the most susceptible (60.73%  ±  6.51 cell viability). On the other hand, it is possible to conclude that concentrations below 0.64 *μ*L/mL are devoid of toxicity, presenting a safety profile for most of the cells studied. Lower concentrations of the oil trigger an increase in resazurin reduction, which may suggest augmentation of the metabolic activity of the cells or a rise in cell proliferation. Further studies should be done to further explore these results. It is, however, important to emphasize that no studies have been previously conducted regarding the cytotoxic effect of* D. carota* subsp.* carota* essential oil. Nevertheless, our group has previously reported that geranyl acetate has very detrimental cytotoxic effects [2].

## 4. Conclusions

This study allowed a better understanding of the bioactivities of* D. carota* subsp.* carota* essential oil. The results showed that this oil had a significant activity towards the inhibition of Gram-positive bacteria,* Cryptococcus neoformans*, and dermatophytes. Importantly, the oil was also efficient in inhibiting the germ tube formation and the preformed biofilms of* Candida albicans*. Despite the oil exhibiting no considerable antiradical activity, it reduced about 20% NO release in LPS-stimulated macrophages, at concentrations devoid of toxicity to these cells. It is reasonable to conclude that concentrations lower than 0.64 *μ*L/mL present a safety profile for different human cell types unveiling the potential application of the essential oil for therapeutical purposes, with a special focus on fungal infections associated with a proinflammatory status. Further experiments disclosing the mechanism of action and* in vivo* tests are of utmost importance to further support the benefit and safety of* D. carota* subsp.* carota* essential oil.

## Figures and Tables

**Figure 1:** Biofilm biomass after treatment with* D. carota* subsp.* carota* essential oil, using the crystal violet assay. Biofilm biomass was determined using the formula (Abs_620_ sample/Abs_620_ control) *∗* 100. Results are shown as mean ± standard deviation of at least three independent determinations carried out in duplicate. ^*∗∗∗*^ *p* < 0.001, ^*∗∗∗∗*^ *p* < 0.0001, compared to control using one-way ANOVA followed by Dunnett's multiple comparison test. Control (100%) corresponds to an absorbance mean value of 1.587.

**Figure 2:** Biofilm viability after treatment with* D. carota* subsp.* carota* essential oil using the XTT viability assay. Results are shown as mean ± standard deviation of at least three independent determinations carried out in duplicate. ^*∗*^ *p* < 0.05, ^*∗∗*^ *p* < 0.01, and ^*∗∗∗*^ *p* < 0.001, compared to control using one-way ANOVA followed by Dunnett's multiple comparison test. Control (100%) corresponds to an absorbance mean value of 0.621.

**Figure 3:** NO scavenging activity of* Daucus carota* subsp.* carota* essential oil. Different concentrations of essential oil (1.25–0.08 *μ*L/mL) were incubated with the NO donor, SNAP (100 mM), in culture medium for 3 h. Results are shown as mean ± SEM of three independent assays, done in duplicate.

**Figure 4:** Anti-inflammatory effect of* Daucus carota* subsp.* carota* in LPS-stimulated Raw 264.7 macrophages: (a) NO production and (b) cell viability. Macrophages were treated with essential oil (1.25–0.08 *μ*L/mL) for 1 h prior to LPS (1 *μ*g/mL) activation and further incubated for 24 h. NO release was determined in the supernatants of the cultures using the Griess reagent (a) and cell viability was assessed on adherent cells using the resazurin reagent and expressed as percentage of cell viability by control cells (b). Results are shown as mean ± SEM of at least three independent assays. (^*∗*^ *p* < 0.05; ^*∗∗*^ *p* < 0.01; ^*∗∗∗∗*^ *p* < 0.0001, compared to LPS). Cell viability control (100%) corresponds to an absorbance mean value of 0.435.

**Table 1:** Composition of the essential oil of *Daucus carota* subsp. *carota*.

RI^a^	RI^p^	Compounds^*∗*^	%
922	1030	*α*-Thujene	t
930	1030	*α*-Pinene	27.2
943	1073	Camphene	0.9
964	1128	Sabinene	0.1
970	1118	*β*-Pinene	4.5
980	1161	Myrcene	2.5
1006	1185	*α*-Terpinene	t
1013	1272	*p*-Cymene	0.1
1020	1206	Limonene	9.0
1025	1235	*Z*-*β*-Ocimene	0.4
1035	1250	*E*-*β*-Ocimene	0.4
1047	1250	*γ-*Terpinene	1.4
1081	1543	Linalool	t
1158	1595	Terpinen-4-ol	0.1
1176	1699	Verbenone	0.1
1233	1838	Geraniol	0.1
1266	1574	Bornyl acetate	0.1
1345	1466	*α*-Longipene	1.0
1362	1753	Geranyl acetate	29.0
1411	1590	*E*-*β*-Caryophyllene	0.4
1443	1660	*α*-Humulene	0.4
1459	2172	(*E*)*-*Methyl isoeugenol	1.4
1466	1699	Germacrene D	0.1
1488	1699	*β*-Himachalene	1.3
1498	1720	*β*-Bisabolene	0.3
1557	1968	Caryophyllene oxide	0.2
1581	2001	Carotol	6.2
1623	2089	11*α*H-Himachal-4-en-1*β*-ol	9.2

		Monoterpene hydrocarbons	46.6
		Oxygen containing monoterpenes	29.5
		Sesquiterpene hydrocarbons	3.5
		Oxygen containing sesquiterpenes	15.6
		Others	1.4

		Total	96.6

^*∗*^Compounds listed in order to their elution on the SPB-1 column.

t: traces (≤0.05%).

RI^a^: retention indices on the SPB-1 column relative to C_8_ to C_24_ *n*-alkanes.

RI^p^: retention indices on the SupelcoWax-10 column relative to C_8_ to C_24_ *n*-alkanes.

**Table 2:** Antibacterial activity (MIC and MLC) of *D. carota* subsp. *carota* essential oil.

Strains	Essential oil		Ampicillin	
	MIC^a^	MLC^a^	MIC^b^	MLC^b^
Gram-positive				
*Bacillus subtilis* ATCC 6633	0.32	0.64	0.06	0.025
*Listeria monocytogenes* CBISA 3183	0.64	>10	2	16
*Staphylococcus aureus* ATCC 6538	0.32	0.64	0.25	0.5
Gram-negative				
*Escherichia coli* ATCC 25922	>10	>10	8	16
*Salmonella typhimurium* ATCC 14028	>10	>10	4	8

MIC and MLC were determined by a macrodilution method and expressed in ^a^ *μ*L/mL and in ^b^ *μ*g/mL.

Results were obtained from three independent experiments performed in duplicate.

**Table 3:** Antifungal activity (MIC and MLC) of *Daucus carota* subsp. *carota* essential oil for *Candida* spp., *Cryptococcus neoformans*, dermatophyte, and *Aspergillus* strains.

Strains	Essential oil		Fluconazole		Amphotericin	
	MIC^a^	MLC^a^	MIC^b^	MLC^b^	MIC^b^	MLC^b^
*Candida albicans *ATCC 10231	5	5	1	>128	NT	NT
*Candida guilliermondii *MAT23	0.32	0.32	8	8	NT	NT
*Candida krusei *H9	5	5	64	64–128	NT	NT
*Candida parapsilosis *ATCC 90018	10	>10	<1	<1	NT	NT
*Candida tropicalis *ATCC 13803	5	>10	4	>128	NT	NT
*Cryptococcus neoformans *CECT 1078	0.16	0.16	16	128	NT	NT
*Epidermophyton floccosum *FF9	0.32	0.32	16	16	NT	NT
*Microsporum canis *FF1	0.64	0.64	128	128	NT	NT
*Microsporum gypseum *CECT 2908	0.64	0.64	128	>128	NT	NT
*Trichophyton mentagrophytes *FF7	0.64	0.64	16–32	32–64	NT	NT
*Trichophyton mentagrophytes *var. *interdigitale *CECT 2958	0.64	1.25	128	≥128	NT	NT
*Trichophyton rubrum *CECT 2794	0.32	0.32	16	64	NT	NT
*Trichophyton verrucosum *CECT 2992	0.64	0.64	>128	>128	NT	NT
*Aspergillus flavus *F44	>10	>10	NT	NT	2	8
*Aspergillus fumigatus *ATCC 46645	2.5	>10	NT	NT	2	4
*Aspergillus niger *ATCC 16404	1.25	>10	NT	NT	1-2	4

MIC and MLC were determined by a macrodilution method and expressed in ^a^ *µ*L/mL and in ^b^ *µ*g/mL.

Results were obtained from three independent determinations performed in duplicate.

**Table 4:** Influence of subinhibitory concentrations of the essential oil of *Daucus carota* subsp. *carota* on germ tube formation of *C. albicans* ATCC 10231.

Essential oil concentration	*Candida albicans *ATCC 10231
(*µ*L/mL)	(% of filamentous cells)
0.00 (control)^a^	100.00 ± 0.00
5.00 (MIC)	0.00 ± 0.00
2.50 (MIC/2)	0.59 ± 1.0
1.25 (MIC/4)	0.88 ± 1.54
0.64 (MIC/8)	1.63 ± 2.82
0.32 (MIC/16)	2.52 ± 4.36
0.16 (MIC/32)	2.90 ± 1.25
0.08 (MIC/64)	21.49 ± 10.89
0.04 (MIC/128)	44.44 ± 8.60
0.02 (MIC/256)	68.54 ± 5.09

^a^Samples with 1% (v/v) DMSO.

**Table 5:** Antioxidant analysis of *D. carota* subsp. *carota* essential oil.

Sample	ABTS^•+a^	ORAC^b^
Essential oil	1924.25	7.13
Trolox	5.53	—

^a^Values expressed as IC_50_ (*µ*g/mL).

^b^Values expressed as *µ*mol TE/mg.

**Table 6:** Effect of *Daucus carota* subsp. *carota* essential oil on cell lines viability.

Essential oil	Macrophages	Epithelial alveolar	Hepatocytes	Keratinocytes
(*µ*L/mL)	Raw 264.7 (%)	cells A549 (%)	HepG2 (%)	HaCaT (%)
0.00 (control)	100 ± 0.0	100 ± 0.0	100 ± 0.0	100 ± 0.0
1.25	9.01 ± 9.01^*∗∗∗*^	64.25 ± 4.66^*∗∗*^	34.54 ± 4.92^*∗∗∗∗*^	55.76 ± 5.03^*∗∗∗∗*^
0.64	92.83 ± 1.04	86.25 ± 5.78	60.73 ± 6.51^*∗∗∗*^	76.30 ± 0.54^*∗∗∗∗*^
0.32	123.60 ± 15.28	110.60 ± 5.72	99.40 ± 5.49	85.21 ± 2.35^*∗∗*^
0.16	141.50 ± 14.56^*∗*^	130.80 ± 9.96^*∗*^	108.80 ± 4.81	94.44 ± 2.94
0.08	154.60 ± 15.55^*∗∗*^	201.90 ± 19.43^*∗∗∗∗*^	122.60 ± 10.43^*∗*^	104.23 ± 2.10

Results expressed as percentage of resazurin reduction compared to control cells maintained in culture medium. Each value represents mean ± SEM of at least three independent experiments done in duplicate. Statistical differences compared to control cells (^*∗*^ *p* < 0.05, ^*∗∗*^ *p* < 0.01, ^*∗∗∗*^ *p* < 0.001, and ^*∗∗∗∗*^ *p* < 0.0001 using one-way ANOVA followed by Dunnett's multiple comparison test).
